# Patient Mix Optimization in Admission Planning under Multitype Patients and Priority Constraints

**DOI:** 10.1155/2021/5588241

**Published:** 2021-03-18

**Authors:** Jialing Li, Li Luo, Guiju Zhu

**Affiliations:** ^1^School of Management, Hunan University of Technology and Business, Changsha 410205, China; ^2^Business School of Sichuan University, No. 24 South Section 1, Yihuan Road, Chengdu, China

## Abstract

Hospital beds are one of the most critical medical resources. Large hospitals in China have caused bed utilization rates to exceed 100% due to long-term extra beds. To alleviate the contradiction between the supply of high-quality medical resources and the demand for hospitalization, in this paper, we address the decision of choosing a case mix for a respiratory medicine department. We aim to generate an optimal admission plan of elective patients with the stochastic length of stay and different resource consumption. We assume that we can classify elective patients according to their registration information before admission. We formulated a general integer programming model considering heterogeneous patients and introducing patient priority constraints. The mathematical model is used to generate a scientific and reasonable admission planning, determining the best admission mix for multitype patients in a period. Compared with model II that does not consider priority constraints, model I proposed in this paper is better in terms of admissions and revenue. The proposed model I can adjust the priority parameters to meet the optimal output under different goals and scenarios. The daily admission planning for each type of patient obtained by model I can be used to assist the patient admission management in large general hospitals.

## 1. Introduction

The balance between the supply and demand of medical resources is a problem faced by the whole world. When a hospital is faced with a discrepancy between supply and demand, it can employ one of two strategies. The first strategy is to expand capacity by increasing staffing or fully developing operating room capabilities; the second is to formulate an admission plan that selects the best mix of patients and gives priority to patients who can be treated effectively. This approach is called patient mix optimization [1]. When the patient mix is combined with the framework of production planning and control, three questions arise. (1) The strategic problem is based on the annual cycle, making decisions about the number of patients to be served each year considering the mix of different types of patients. (2) The decision cycle of the tactical layer is generally from month to week. (3) The operation layer is mainly involved in the determination of the patients to be served every day and when they enter the hospital [2]. These decisions are aimed towards allocating different types of patients to resources involved in inpatient services.

As the demand for medical resources increases year by year, the unlimited expansion of capacity is not possible, especially in the context of China's medical system. The medical resources of China's large general hospitals are often overloaded. The bed utilization rate of public tertiary hospitals in China in 2019 was as high as 97.5%. In our hospital, due to the long-term addition of beds, the bed utilization rate in some departments exceeded 100% [3].

In China, large general hospitals mainly provide medical services for acute, severe, and complex diseases, and community hospitals are used to treat chronic and mild diseases. However, due to the absence of a gatekeeper system, Chinese patients are free to choose which hospitals to attend for treatment. Patients tend to go to large hospitals first, rather than to community hospitals. As a result, large hospitals are often overcrowded, while the medical resources of primary hospitals are relatively idle. According to the data of the *2019 China Health and Family Planning Development Bulletin* published by the National Health Planning Commission, the number of admissions to tertiary hospitals increased from 92.92 million in 2018 to 104.83 million in 2019, while the number of admissions to primary health care institutions decreased from 43.76 million to 42.95 million [4].

Therefore, for large general hospitals in China in which resources have been overloaded and cannot increase rapidly in the short term, formulation of an admission plan can alleviate the mismatch between supply and demand. The goal of admission planning is to achieve an acceptable match between demand and capacity, to improve the efficiency of high-quality medical services. From a demand perspective, when a large number of inpatients cannot be admitted due to the scarcity of hospital beds, a feasible solution is to give priority to patients who need more inpatient services [5]. This arrangement not only ensures the fairness of the distribution of medical resources but also reduces the waste of high-quality resources and improves resource utilization. For hospitals, the matching of demand and capacity is important. When general hospitals face different admission needs, they can optimize admission planning by constructing a mathematical planning model which optimizes the allocation of limited medical resources. This problem is the focus of this article.

This paper is relevant to the current literature from two perspectives. The first is that we conducted research into the combination of patient mix with resource scheduling. Part of the literature focuses on the follow-up scheduling of medical resources by introducing the concept of patient mix. Patient mix involves dividing patients into several categories and then assigning patients to different follow-ups, a situation which belongs to the scope of hospital operation management. This type of literature primarily includes research into resource scheduling optimization for multipriority patients [6]. Meisami et al. [7] used mortality risk-based metrics and a data-driven mixed integer model to conduct research into patient admission management in intensive care units. Roshanaei et al. [8] developed the first exact decomposition approaches for multilevel operating room planning and scheduling that integrates case mix planning, master surgical scheduling, and surgery sequencing in the presence of multiple surgical specialties.

The second is the research status of admission planning. Part of the literature is concerned with the number of patients and the optimization of patient mix from a tactical and strategic level, to assist the hospital in determining the best mix of admitted patients, thereby improving the utilization of medical resources. The main problem is patient admission planning, including ensuring an optimal patient mix, which matches available capacity with demand. This type of patient admission planning includes the selection of the best patient mix and the matching of available capacity and demand [9, 10]. Adan and Vissers [11] conducted a study on the best way in which to formulate admission planning to meet patient throughput and maximize resource utilization when capacity is limited. Their study was the earliest investigation into patient admission planning. Later, stochastic resource requirements were considered in further research into patient admission planning [12]. Since then, many scholars have conducted studies into patient admission planning [13–15]. Ma and Demeulemeester [16] proposed a comprehensive multilevel approach to the study of a hospital's patient mix and capacity planning, to improve resource efficiency and improve patient service. Their method addresses three aspects: the case mix, main surgery scheduling, and performance evaluation. Freeman et al. [17] developed a multiphase approach that utilizes mathematical programming and simulation to generate a pool of candidate solutions for case mix planning. McRae and Brunner [18] formulated a mixed integer programming model for case mix planning, with different stochastic and deterministic extensions.

In summary, the main contributions of this article to the current literature are as follows:

- The introduction of constraints with which to prioritize patients. Most current admission management studies only consider a single medical resource [19, 20]. Based on data from large general hospitals in China, this paper introduces constraints that can quantify the priority of patients. This article also considers the tactical issue of how to execute reasonable admission planning for a hospital through patient mix optimization when the hospital encounters patient groups with different priorities, to ensure effective use of multiple medical resources
- The model is flexible and adaptable and can be dynamically adjusted. Although the management of admission planning has received tremendous attention, in terms of practicality, some models are subject to specific assumptions, and the applicability of those studies needs to be strengthened [21–23]. Taking into account the differences in the characteristics and resource consumption of different types of patients, this paper describes the construction of a mathematical planning model with multitype patients and priority constraints to generate an optimal plan for patient admission. Through sensitivity analysis, we have obtained results in different scenarios. Different types of hospitals can assist patient admission management according to their actual conditions by personalizing the parameters such as the upper and lower bounds of priority weight, priority score, and target resource utilization
- The patient admission planning in this article is a follow-up study based on data-driven patient classification. The current mainstream method abroad is to develop a scoring system for specific diseases and then apply it to patient prioritization [24, 25]. However, due to the imperfect indicators of this method, the results may be biased in determining the priority of patients. Data-driven demand classification has become a new research trend [26–28]. The patient types in this article are based on our previous research results. The study uses the patient's admission information as input and incorporates machine learning methods to build classification models and scientifically classifies the preadmission elective patients [29]

The remainder of this paper is structured as follows. In Section 2, we describe the background of the research.  Section 3 builds the model of admission planning for elective patients. In Section 4, a case study is described, and the sensitivity analysis and model comparison analysis are described in Section 5. In the final section, a conclusion is drawn.

## 2. Problem Description

In this section, we consider the patient admission planning of large general hospitals under China's national conditions, in order to provide policy recommendations for the hospital's tactical decision-making. The problems considered in this paper are described as follows.

### 2.1. Background

West China Hospital (WCH) is a large tertiary hospital in China, which has totally 4300 beds and 43 specialized units. WCH is a national-level treatment center for intractable diseases, but the waiting list for elective patients, who could have been treated in community hospitals, also sought admission into general hospitals. To a certain extent, such patients occupy the admission quota of patients with severe illness, which further aggravates the imbalance between supply and demand of admission services in general hospitals. WCH is a typical and representative tertiary hospital in China. The above issue that this article focuses on is also the common challenge faced by other large tertiary hospitals. This article chooses WCH as a research case to study such major research question: how to reasonably allocate high-quality resources among different types of patients.

### 2.2. Research Question and Purpose

We abstract the abovementioned practical problems as part of patient admission planning. In this paper, the issue of admission planning of elective patients refers to the decision on the number of elective patients and the best mix of patients with different priorities given the constraints of access to medical resources. The objective of this study is to generate an optimal admission plan of elective patients with stochastic length of stay and the resource consumption of each type of patients.

The uniqueness of this article is reflected in three aspects. (1) Considering multiple medical resource constraints: the resources included are hospital beds, medical examination resources, and nursing resources. They are considered as the most critical for the problem due to limitations in availability. (2) Data-driven patient classification: based on previous research results [29], according to the patient's disease health status, type of medical insurance, location, and other personal information, machine learning methods can be used to predict the probability of patients waiting to be admitted. The authors of that article divide patients into three categories based on the probability by the machine learning algorithm: probability of admission to type I *p* ∈ [0.8, 1], probability of admission to type II *p* ∈ (0.5, 0.8), and probability of admission to type III *p* ∈ [0, 0.5]. (3) Introducing patient priority constraints of large hospitals under China's national conditions: heterogeneity of patients implies that there are different groups of patients, each with their own resource requirements, length of stay, and unit revenue. We assign different priority scores to different types of patients. The higher the admission priority, the higher the score. The priority of each type of patient is no longer subdivided internally, that is, the same type of patient is given a uniform score.

### 2.3. Optimization Process

The objective function is to maximize revenue, while considering the deviation cost of resource utilization. Given the ideal target capacity of each medical resource, an integer programming model can be constructed to determine the number of patients admitted to the hospital and the mix of different types of patients in the cycle. The best patient mix depends upon the characteristics of the patient type and the amount of medical resources available to the department.

### 2.4. Expected Results

The result produced by this model is a tactical hospital admission planning, which describes the number of hospitalized patients and the proportion of different types of patients during the planning cycle. It can be dynamically adjusted according to the expected utilization of different medical resources involved. Admission planning can be used to guide the hospital admission arrangements for daily operation. The structure of the admission planning for elective patients with multiple priority is shown in Figure 1.

## 3. The Proposed Mathematical Model

In this section, we explain the notation used in the model and then present an admission planning model that considers multiple types of patients and their priority constraints.

### 3.1. Sets

*I*: Set of patient types, *i* ∈ *I*,

*T*: Set of days in planning circle, *T* = {1, 2, ⋯, *τ*}, *t* ∈ *T*, *τ* = 28, the planning cycle for this article is 28 days,

*R*: Set of medical resources, *R* = {1, 2, 3}, *r* ∈ *R*,

*r* = 1: Bed resources,

*r* = 2: Medical examination resources,

*r* = 3: Nursing resources.

### 3.2. Parameters

*r*_*i*_: Revenues generated by treated a patient from type *i*,

*n*: The total estimated number of patients admitted in a planning cycle,

*e*_*i*_: The time required for a patient from type *i* to perform medical technical examination (cases/hours),

*n*_*i*_: The nursing workload (in hours) required for a patient from type *i* (the higher the priority, the greater the nursing workload),

*P*_*it*_: Probability that the length of stay is *t* days of a patient from type *i*,

${\tilde{P}}_{\text{is}}$: Probability that the length of stay is over *s* days of a patient from type *i*,

*s*_*i*_: Priority score of patients from type *i*,

*L* ^*p*^: Lower bound of average priority weight for patients

*α*_*i*_: Lower bound of admission proportion of patients in type *i*,

*β*_*i*_: Upper bound of admission proportion of patients in type *i*,

*AC*_*rt*_: Available capacity of resource *r* on day *t*,

*TC*_*rt*_: Target capacity of resource *r* on day *t*,

*c*_*r*_^+^: Positive deviation cost of resource *r*,

*c*_*r*_^−^: Negative deviation cost of resource *r*.

### 3.3. Decision Variables

*x*_*it*_: Number of patients from type *i* admitted on day *t* of the planning cycle.

The following indirect variables are directly related to the decision variables *x*_*it*_:

*M*_*it*_: Indirect variables, the total number of patients from type *i* on day *t*,

*C*_*rt*_^+^: Auxiliary variable, excess capacity of resource *r* on day *t*,

*C*_*rt*_^−^: Auxiliary variable, spare capacity of resource *r* on day *t*,

*θ*_*i*_: Admission ratio (unit: %) of the patients from type *i*, it can be understood as the percentage of each type of patient to the total planned admissions, which can be obtained by *x*_*it*_ :  *θ*_*i*_ = ∑_*t*=1_^*T*^*x*_*it*_/∑_*t*=1_^*T*^∑_*i*=1_^*I*^*x*_*it*_.

### 3.4. Objective Function

Given the above parameter information, how does the hospital generate an appropriate admission plan? The model constructed in this article is organized as follows.

First of all, the objective function of the model is the maximum profit, as shown in

(1) $$\begin{array}{c} \mathrm{Max}Z=\overset{I}{\underset{i=1}{\sum }}\overset{T}{\underset{t=1}{\sum }}r_{i}x_{it}-\overset{R}{\underset{r=1}{\sum }}\overset{T}{\underset{t=1}{\sum }}c_{r}^{+}C_{rt}^{+}-\overset{R}{\underset{r=1}{\sum }}\overset{T}{\underset{t=1}{\sum }}c_{r}^{-}C_{rt}^{-}. \end{array}$$

The objective function (1) is described from the perspective of revenue and cost of resource utilization. The hospital accepts a patient from type *i* which will generate certain benefits. When the hospital's resources are underutilized or overused, it brings additional costs, as shown in Figure 2.

There may be two situations between the target capacity and the actual capacity. One is when the actual capacity exceeds the target capacity, so the capacity is overutilized, which we call positive deviation. If the actual capacity is lower than the target capacity, there will be underutilized resources, which we call negative deviation.

It should be noted that the revenues discussed in this paper are related to the criticality of the patient, the rate of disease recovery after treatment, and the contribution to the value of the subject. The setting of revenue parameters is not only for economic considerations but also includes other factors such as broad social influences. It is a modified price. We assume that the revenues of serving patients with intractable diseases are higher than those of ordinary patients. This is not only because of the cost of their diagnosis and treatment but also because the service of critically ill patients is more in line with the positioning of a general hospital and contributes to the development of clinical disciplines.

In summary, setting the objective function to maximize revenue is to use price tools in economics to regulate the process of resource allocation to optimize efficiency. It is also the choice to maximize resource efficiency after considering moral and social factors.

### 3.5. Restrictions

Hospital beds are limited. Therefore, the total number of patients that can be admitted to the hospital during cycle *T* needs to be restricted. Constraint (2) means that the number of admissions for all types of patients is less than the estimated total number of admissions during the *T* cycle.

(2) $$\begin{array}{c} \overset{I}{\underset{i=1}{\sum }}\overset{T}{\underset{t=1}{\sum }}x_{it}\leq n. \end{array}$$

In this article, we assume that the hospital divides patients into *i* types according to the probability of admission. In order to meet the positioning of a general public hospital, it is necessary to restrict the admission proportion of different types of patients. Constraint (3) and constraint (4) stipulate the upper and lower bounds of the admission proportion of patients from type *i* in the *T* cycle.

(3) $$\begin{array}{c} \overset{T}{\underset{t=1}{\sum }}x_{it}\leq \beta_{i}\overset{I}{\underset{i=1}{\sum }}\overset{T}{\underset{t=1}{\sum }}x_{it},\;\forall i\in I,\forall t\in T, \end{array}$$

(4) $$\begin{array}{c} \overset{T}{\underset{t=1}{\sum }}x_{it}\geq \alpha_{i}\overset{I}{\underset{i=1}{\sum }}\overset{T}{\underset{t=1}{\sum }}x_{it},\;\forall i\in I,\forall t\in T. \end{array}$$

Since different types of patients get different admission scores, the higher the priority, the higher the score. We also set a minimum average priority score for all types of patients admitted to the hospital. Constraint (5) means that the average priority score of all admitted patients in the hospital should meet at least a certain lower bound to meet the needs of patients with intractable diseases.

(5) $$\begin{array}{c} \overset{I}{\underset{i=1}{\sum }}s_{i}\left(\overset{T}{\underset{t=1}{\sum }}x_{it}\right)\geq L^{p}\cdot \overset{I}{\underset{i=1}{\sum }}\overset{T}{\underset{t=1}{\sum }}x_{it}. \end{array}$$

We use probability to indicate the length of stay. Different types of patients have different distributions of length of stay, which follow discrete distributions. For patients from type *i*, suppose the shortest length of stay is 1 day, and the longest hospital stay is 28 days. Let *P*_*it*_ denote the probability that the actual length of stay for the patient from type *i* is *t* days. When the patient's length of stay exceeds *s* days (*s* ∈ {0, ⋯, *T* − 1}), the cumulative probability distribution, ${\tilde{P}}_{\text{is}}$, can be calculated and used to express the probability that the length of stay for the patient from type *i* exceeds *s* days after admission. The distribution of length of stay and cumulative length of stay for a patient of type *i* can be described as Table 1, and the conversion relationship between *P*_*it*_ and ${\tilde{P}}_{\text{is}}$ is summarized as ${\tilde{P}}_{\text{is}}=1-\sum_{t=0}^{s}P_{it}$, *s* ∈ {0, ⋯, *T* − 1}. Specific information is shown in Table 1.

Based on the principles discussed above, the intermediate variable *M*_*it*_ can be calculated to indicate the number of patients in the hospital on day *s* of type *i*, expressed as constraint (6). Constraint (7) means that the actual utilization of the hospital bed in the *T* period cannot exceed its available capacity.

(6) $$\begin{array}{c} M_{it}=\overset{t-1}{\underset{s=0}{\sum }}{\tilde{P}}_{\text{is}}\cdot x_{it},\;\forall i\in I,t\in T, \end{array}$$

(7) $$\begin{array}{c} \overset{I}{\underset{i=1}{\sum }}M_{it}\leq {AC}_{rt},\;\forall t\in T,r=1. \end{array}$$

Constraint (8) and constraint (9) require that the actual capacity used of inspection resources and nursing resources cannot exceed the available capacity during the *T* period.

(8) $$\begin{array}{c} \overset{I}{\underset{i=1}{\sum }}e_{i}x_{it}\leq {AC}_{rt},\;\forall t\in T,r=2, \end{array}$$

(9) $$\begin{array}{c} \overset{I}{\underset{i=1}{\sum }}n_{i}M_{it}\leq {AC}_{rt},\;\forall t\in T,r=3. \end{array}$$

Constraints (10)–(12) are descriptions of auxiliary variables *C*_*rt*_^+^, which represent the excess capacity (positive deviation) between the actual capacity of each resource and the target capacity per day. Constraints (13)–(15) are descriptions of auxiliary variables *C*_*rt*_^‐^, which represent the idle capacity (negative deviation) between the target capacity of each resource and the actual capacity used each day. Constraint (16) requires the decision variable to be a positive integer.

(10) $$\begin{array}{c} C_{rt}^{+}={\left(\overset{I}{\underset{i=1}{\sum }}M_{it}-{TC}_{rt}\right)}^{+},\;\forall t\in T,r=1, \end{array}$$

(11) $$\begin{array}{c} C_{rt}^{+}={\left(\overset{I}{\underset{i=1}{\sum }}e_{i}x_{it}-{TC}_{rt}\right)}^{+},\;\forall t\in T,r=2, \end{array}$$

(12) $$\begin{array}{c} C_{rt}^{+}={\left(\overset{I}{\underset{i=1}{\sum }}n_{i}M_{it}-{TC}_{rt}\right)}^{+},\;\forall t\in T,r=3, \end{array}$$

(13) $$\begin{array}{c} C_{rt}^{-}={\left({TC}_{rt}-\overset{I}{\underset{i=1}{\sum }}M_{it}\right)}^{+},\;\forall t\in T,r=1, \end{array}$$

(14) $$\begin{array}{c} C_{rt}^{-}={\left({TC}_{rt}-\overset{I}{\underset{i=1}{\sum }}e_{i}x_{it}\right)}^{+},\;\forall t\in T,r=2, \end{array}$$

(15) $$\begin{array}{c} C_{rt}^{-}={\left({TC}_{rt}-\overset{I}{\underset{i=1}{\sum }}n_{i}M_{it}\right)}^{+},\;\forall t\in T,r=3, \end{array}$$

(16) $$\begin{array}{c} x_{it}\in \left\{0,1,2,\cdots ,n\right\},\;\forall i\in I,\;\forall t\in \left\{1,\cdots ,T\right\}. \end{array}$$

Finally, the integer programming model of this article is summarized as follows:

(17) $$\begin{array}{c} \mathrm{Max}Z=\overset{I}{\underset{i=1}{\sum }}\overset{T}{\underset{t=1}{\sum }}r_{i}x_{it}-\overset{R}{\underset{r=1}{\sum }}\overset{T}{\underset{t=1}{\sum }}c_{r}^{+}C_{rt}^{+}-\overset{R}{\underset{r=1}{\sum }}\overset{T}{\underset{t=1}{\sum }}c_{r}^{-}C_{rt}^{-}\\ \text{s}.\text{t}.\;\overset{I}{\underset{i=1}{\sum }}\overset{T}{\underset{t=1}{\sum }}x_{it}\leq n\\ \;\overset{T}{\underset{t=1}{\sum }}x_{it}\leq \beta_{i}\overset{I}{\underset{i=1}{\sum }}\overset{T}{\underset{t=1}{\sum }}x_{it},\;\forall i\in I,\forall t\in T\\ \;\overset{T}{\underset{t=1}{\sum }}x_{it}\geq \alpha_{i}\overset{I}{\underset{i=1}{\sum }}\overset{T}{\underset{t=1}{\sum }}x_{it},\;\forall i\in I,\forall t\in T\\ \;\overset{I}{\underset{i=1}{\sum }}s_{i}\left(\overset{T}{\underset{t=1}{\sum }}x_{it}\right)\geq L^{p}\cdot \overset{I}{\underset{i=1}{\sum }}\overset{T}{\underset{t=1}{\sum }}x_{it}\\ \;M_{it}=\overset{t-1}{\underset{s=0}{\sum }}{\tilde{P}}_{\text{is}}\cdot x_{it},\;\forall i\in I\\ \;\overset{I}{\underset{i=1}{\sum }}M_{it}\leq {AC}_{rt},\;\forall t\in T,r=1\\ \;\overset{I}{\underset{i=1}{\sum }}e_{i}x_{it}\leq {AC}_{rt},\;\forall t\in T,r=2\\ \;\overset{I}{\underset{i=1}{\sum }}n_{i}M_{it}\leq {AC}_{rt},\;\forall t\in T,r=3\\ \;C_{rt}^{+}={\left(\overset{I}{\underset{i=1}{\sum }}M_{it}-{TC}_{rt}\right)}^{+},\;\forall t\in T,r=1\\ \;C_{rt}^{+}={\left(\overset{I}{\underset{i=1}{\sum }}e_{i}x_{it}-{TC}_{rt}\right)}^{+},\;\forall t\in T,r=2\\ \;C_{rt}^{+}={\left(\overset{I}{\underset{i=1}{\sum }}n_{i}M_{it}-{TC}_{rt}\right)}^{+},\;\forall t\in T,r=3\\ \;C_{rt}^{-}={\left({TC}_{rt}-\overset{I}{\underset{i=1}{\sum }}M_{it}\right)}^{+},\;\forall t\in T,r=1\\ \;C_{rt}^{-}={\left({TC}_{rt}-\overset{I}{\underset{i=1}{\sum }}e_{i}x_{it}\right)}^{+},\;\forall t\in T,r=2\\ \;C_{rt}^{-}={\left({TC}_{rt}-\overset{I}{\underset{i=1}{\sum }}n_{i}M_{it}\right)}^{+},\;\forall t\in T,r=3\\ \;x_{it}\in \left\{0,1,2,\cdots ,n\right\},\;\forall i\in I,\forall t\in \left\{1,\cdots ,T\right\}. \end{array}$$

## 4. Case Study

The numerical experiment was performed using an Intel® Core™ i7-7700 CPU@3.60 GHz, 3.6 Gb. We used the optimization software ILOG CPLEX12.8 to solve the exact solution of the mixed integer linear programming model.

We hoped to achieve the following goals through case analysis: (1) determine the optimal patient mix for the department to maximize the revenue, (2) analyze the impact of different patient mixes and medical resources on revenue and admissions, and (3) evaluate admission planning strategies under different scenarios to provide recommendations for the hospital.

### 4.1. Parameter Settings

The parameters were derived from historical data from the Department of Respiratory Medicine of WCH. The respiratory department has a total of 290 beds. The working hours of the examination equipment, doctors, and nurses are eight hours per day, and the planned time interval was 28 days. The proportion of emergency to elective patients in the respiratory medicine department of WCH was 1 : 2. Considering a reservation strategy for emergency patients, we reserved 30% of the capacity for emergency admissions, based on the proportion of patients. The contribution of the hospital includes not only the benefits of diagnosis and treatment but also the contribution to the development of the discipline during the treatment process. Therefore, the higher the priority, the higher the benefit to the hospital for patients. For specific parameter settings, see Tables 2–4.

### 4.2. Results

In this section, we present the results of a four-week patient admission planning using the model, as shown in Figure 3. Because the model restricts the admission proportion and priority of each type of patient, the total number of patients of type I is more than those of type II, and type II has more patients than type III. The objective function of the model is 6462.4. The total number of admissions is 570, of which the number of admissions of the three types of patients and their proportions are 399 (70%), 114 (20%), and 57 (10%), respectively.

## 5. Discussion

### 5.1. Sensitivity Analysis

Sensitivity analysis was used mainly to observe the impact of changes in the decision-making environment on the results. The decision-making environment here is a parameter that is prone to change in practice. In this section, we analyze the results from three aspects: unit resource consumption, priority constraints, and target capacity changes. The sensitivity analysis is carried out from the following four perspectives.

#### 5.1.1. Impact of Nursing Capacity on Outcomes

Resource consumption mostly involves changes in the length of stay, changes in the time of medical examinations, and the workload of nursing care. Because the length of stay in this paper is expressed as a probability, it is inherently random, so this article takes the nursing duration parameter as an example for sensitivity analysis. The medical examinations can refer to the change of nursing duration and so will not be repeated.

The nursing time of the three types of patients set by the basic model is 1.5, 1, and 0.5 hours, respectively. Scenarios 1–3 are aimed at adjusting the parameters of nursing time of type I, after fixing the unit nursing time of type II and type III. Similar processing for scenarios 4–6 and scenarios 7–9 adjusts the parameters of the unit nursing time of type II and type III.

From Table 5 and Figure 4, the following can be seen:

1. In scenarios 1–3, compared with the results of the benchmark parameters (scenario 2), after increasing the length of care for the first type of patients, the number of admissions decreases, and the income slightly decreases. Scenario 3 reflects the situation when the length of care for the first type of patients is reduced, the number of admissions showed an upward trend, but the income declined
2. In scenarios 4–6, after increasing the length of care for patients in type II, compared with the results of the benchmark parameter (scenario 5), the number of admissions and benefits of scenario 4 have increased. Scenario 6 reduces the length of care for patients in type II, the number of admissions remained unchanged, but the income dropped slightly
3. In scenarios 7–9, compared with the results of the benchmark parameter (scenario 8), when the length of the third type of nursing is increased, the benefits and the total number of admissions increase; when the length of the third type of nursing is reduced, the income and the total number of admissions have increased slightly

#### 5.1.2. Impact of Admission Proportion on Outcome

The admission proportion of each type of patient is restricted by the parameters *α*_*i*_ and *β*_*i*_ to control the upper and lower bounds.  Table 6 shows the changes in *α*_*i*_ and *β*_*i*_ when other parameters remain unchanged. We can use this as the input for sensitivity analysis.

From Figure 5, the following can be seen:

1. In scenarios 1–3, after gradually reducing the upper bound of the admission proportion of type I, the income and the total number of admissions show a downward trend
2. In scenarios 4–6, after gradually changing the lower bound of the admission proportion of type I, the income and the total number of admissions show an upward trend. The upper bound increases, and the proportion of patients of type I also increases. Patients of type I in scenarios 1, 2, and 3 are 89.76%, 79.93%, and 70.00%, respectively, while type I in scenarios 4–6 has always been 70%. That is, the adjustment of the upper bound has a significant influence on the result, while the influence of the lower bound has little influence on the result
3. Scenarios 6–8 increase the upper bound of the second type of patients. Although the total number and income have not changed much, the proportion of patients has changed. The first type of patients remains at 69%, while the rate of admission to type II decreases as the upper bound decreases. Scenarios 8 and 9 have similar results

#### 5.1.3. Impact of Priority Score on Outcome

The priority score of the patient is an important factor in the admission process. By giving the lowest average priority score, the admission level of the entire hospital is constrained. Since formulas (3) and (4) impose hard constraints on the admission proportion of each type of patient, we remove constraints (3) and (4) to discuss the results caused by changes in priority scores, as shown in Figure 6. The results are as follows:

1. Because there is no hard constraint on the admission proportion of each type of patient, overall, the outcome and the number of admissions have increased, and the unit revenue of the first type of patient is the highest, Therefore, the model is more inclined to treat the first type of patients, which can account for 99%
2. As the lower bound of the priority score gradually increases, the proportion of the number of admissions from type I gradually increases. When the average priority score of the admitted patients is at least 9 points, all of the admitted patients are from type I. Specifically, 3 points and 8 points are important threshold. When the score is 1 to 3, there is no change in the results. Using 3 points as the critical value, when the priority score increases to 4 to 8, the proportion of patients in type I further increases. At this time, the revenue increases slightly, but when the score is increased to 9 points, the hospital only admits patients of type I

The above results show that the setting of priority scores cannot be increased indefinitely and should be set according to the actual situation of the hospital.

#### 5.1.4. Impact of the Adjustment of the Target Capacity on the Result

We explored different values of the target capacity to observe the effect on the results. Scenarios 1–7 in Table 7 are the optimal solutions when the target utilization of resources is 90%, 91%, 92%, 93%, 94%, 95%, and 96%, respectively.

From Figure 7, it can be seen that, as the target capacity increases, the utilization rate of resources also increases. At this time, the hospital's revenue first declines and then rises as the target capacity increases. It means that the more the target production capacity, the better the effect. It is necessary to make rational use of resources to avoid idleness or underutilization.

### 5.2. Comparison with Model II

We compared model I, which uses the priority constraints proposed in this paper, with model II. Model II eliminates the restriction on the proportion of each type of patient in the cycle, as described in formulae (3) and (4). The restriction on the priority of the patients is according to formula (5), and patients are homogenized. Model II is a simplified model after removing the priority constraints in model I. The details of the difference between models I and II are shown in Table 8.

A comparative analysis of model I and model II was carried out to evaluate the advantages and effectiveness of model I, as proposed in this paper. The results of model II and model I under the three scenarios can be seen in Table 9 and Figures 8 and 9.

1. Admissions: without priority constraints, the total number of patients in model II was 570. The admissions in model I in scenarios 1, 2, and 3 were 586, 583, and 500, respectively. The admission proportions in scenario 1 were 89.76%, 10.07%, and 0.17%, respectively, while those of scenario 2 were 69.64%, 29.33%, and 1.03% and those of scenario 3 were70.00%, 20.00%, and 10.00%, respectively
2. Objective function: without the constraint of priority, the revenue of model II was 6462.4. The objective function values of the three scenarios of model I were 7138.1, 6815.55, and 6673.95
3. Patient admission status: we found that in model I under the three scenarios, the total number of patient and revenue were better than model II without priority. ① Patients in model I are heterogeneous. Taking scenario 3 as an example, we plotted the admission status of each type of patient every day, as shown in Figure 9. The model assumes that the initial state of the hospital is empty and admits patients. Because of the priority constraints, the admission curves of the three types of patients in the figure are admitted strictly in accordance with the constraints. Model I admits patients according to the severity of the patient's disease. The hospital's goals can be achieved by adjusting the admission proportion of each type of patient. ② The patients in model II are homogeneous, and there is no subdivision, so there is only an independent curve to represent the number of admissions per day. Model II admits patients according to the first-come, first-served rule. In a relatively average situation, more patients are admitted
4. Application scenario: in the results of model I, the first type of patients accounts for a higher proportion (at least 50% or more), and the third type of patients accounts for a smaller proportion. Therefore, the results of model I are more in line with the positioning of a general hospital. Model II is more suitable for community hospitals that are not sensitive to patient types

The insights into management obtained from the above results are as follows:

1. There is a trade-off between admissions and revenue. If the hospital wants as many admissions as possible, it will need to treat more patients of type III and sacrifice the number of patients in type I. Because patients of type I occupy more medical resources, although their unit income is more than other types of patients, type III patients often occupy fewer beds and nursing resources, and their turnover rate is higher, so more type III patients can be admitted at the same time. Compared with type I patients, the patients of type III create more benefits
2. China's public general hospitals do not always take revenue as the most important goal. In order to balance income and the treatment of critically ill patients, efficient and reasonable use of high-quality medical resources in general hospitals is the key issue. For general hospitals, the revenue lies not only in economic profit but also in the patient's contribution to scientific research, discipline development, and other aspects. Therefore, for general hospitals in China, the benefit is not the more the better. However, it is important to determine reasonable admission proportions for different types of patients under the condition of ensuring a certain benefit, to ensure that high-quality medical resources are matched with high-quality patients

## 6. Conclusions

The optimization of patient mix has become an important tool for hospital management. By planning and arranging admissions for different types of patients, this approach can effectively guide the admission of patients with daily operations. This paper discusses the best way in which to obtain optimal admission planning through patient mix optimization when the hospital's medical resource capacity is limited in a certain planning cycle, so as to achieve specific resource utilization goals and maximize revenue when faced with different types of patients. The main conclusions are as follows:

1. The consumption of medical resources will cause changes in the total number of patients and income. It is necessary to formulate a reasonable unit resource consumption to avoid underutilization or overuse of resources
2. The admission proportion and priority score are important constraints, which are not as high as possible. Hospital managers should determine a reasonable upper and lower bound for proportions and priority scores, based on the expected goals
3. Model I can adjust the priority parameters to meet the optimal output under different goals and scenarios. Therefore, compared with model I, the revenue and admissions of model II are lower than model I

In the future, we shall investigate the patient mix optimization under more complex situation, such as the arrival of emergency patients and overutilization of medical resources. In particular, this study provides a research basis for further research on the admission planning issue of how to match infected patients of different severity with limited medical resources during the COVID-19 pandemic. Applying the patient mix optimization in this article to the scenario of COVID-19 pandemic is a good research direction.

## Figures and Tables

**Figure 1:** Structure of the admission planning of elective patients.

**Figure 2:** The relationship between actual capacity used and target capacity.

**Figure 3:** Number of admissions for multitype patients.

**Figure 4:** The impact of changes in nursing capacity consumption on outcome.

**Figure 5:** Outcome under different admission proportions.

**Figure 6:** Impact of priority scores on outcome.

**Figure 7:** Outcomes under different target capacity.

**Figure 8:** Results of model I under three scenarios and model II.

**Figure 9:** Daily admissions for model I and model II.

**Table 1:** Description of the distribution of LOS and cumulative LOS of patients from type *i*.

*t*	1	2	3	…	*T*
*P*_*it*_	*P*_*i*1_	*P*_*i*2_	*P*_*i*3_	…	*P*_*it*_
*s*	0	1	2	…	*T* − 1
${\tilde{P}}_{\text{is}}$	1	$1-\left({\tilde{P}}_{i1}+{\tilde{P}}_{i2}\right)$	$1-\left({\tilde{P}}_{i1}+{\tilde{P}}_{i2}\right)$	…	$1-\sum_{t=0}^{s}{\tilde{P}}_{it}$

**Table 2:** Cumulative probability distribution ${\tilde{P}}_{\text{is}}$ of length of stay in the three types of patients.

*s*	Type I	Type II	Type III
0	1	1	1
1	0.99	0.99	0.99
2	0.98	0.98	0.98
3	0.97	0.97	0.97
4	0.95	0.96	0.93
5	0.91	0.94	0.9
6	0.85	0.88	0.83
7	0.77	0.79	0.72
8	0.68	0.7	0.64
9	0.61	0.64	0.63
10	0.54	0.58	0.57
11	0.48	0.51	0.48
12	0.41	0.44	0.46
13	0.34	0.36	0.39
14	0.27	0.29	0.3
15	0.23	0.25	0.27
16	0.2	0.22	0.24
17	0.17	0.19	0.21
18	0.14	0.16	0.17
19	0.12	0.14	0.15
20	0.1	0.12	0.13
21	0.08	0.1	0.1
22	0.07	0.08	0.09
23	0.06	0.07	0.07
24	0.05	0.05	0.06
25	0.04	0.04	0.05
26	0.03	0.03	0.04
27	0.02	0.02	0.03

**Table 3:** Parameters related to patients.

	Type I	Type II	Type III
*r*_*i*_	170	160	150
*e*_*i*_	1.5	1	1.5
*n*_*i*_	1.5	1	0.5
*s*_*i*_	9	6.5	3
[*α*_*i*_, *β*_*i*_]	[0.7, 0.5]	[0.2, 0.1]	[0.1, 0]

**Table 4:** Parameters related to medical resources.

Medical resources	*ACr*	*TCr*	*c*_*r*_^+^	*c*_*r*_^−^
Hospital bed	203	183	20	30
Medical examination	201.6	181	20	30
Nursing	561	512	20	30

**Table 5:** Value of objective function under the change of nursing capacity.

Scenario	Type I	Type II	Type III	Revenue	Admissions
1	1.75	1	0.5	6418.4	550
2	1.5	1	0.5	6462.4	570
3	1.25	1	0.5	6311.9	580
4	1.5	1.25	0.5	6745	580
5	1.5	1	0.5	6462.4	570
6	1.5	0.75	0.5	6415	570
7	1.5	1	0.75	6684	580
8	1.5	1	0.5	6462.4	570
9	1.5	1	0.25	6837	580

Note: scenarios 2, 5, and 8 are the benchmark parameters of the model.

**Table 6:** Parameter settings of admission proportion.

Scenarios	High (*α*_1_, *β*_1_)	Middle (*α*_2_, *β*_2_)	Low (*α*_3_, *β*_3_)
1	(0.9, 0.5)	(0.2, 0.1)	(0.1, 0)
2	(0.8, 0.5)	(0.2, 0.1)	(0.1, 0)
3	(0.7, 0.5)	(0.2, 0.1)	(0.1, 0)
5	(0.7, 0.6)	(0.2, 0.1)	(0.1, 0)
6	(0.7, 0.4)	(0.2, 0.1)	(0.1, 0)
7	(0.7, 0.5)	(0.4, 0.1)	(0.1, 0)
8	(0.7, 0.5)	(0.3, 0.1)	(0.1, 0)
9	(0.7, 0.5)	(0.2, 0.1)	(0.2, 0)
10	(0.7, 0.5)	(0.3, 0.1)	(0.1, 0.05)

Note: scenario 3 is the benchmark parameter.

**Table 7:** Results under different target capacities.

Scenario	Target capacity	Proportion	Revenue	Admissions
1	183	90%	6462.4	570
2	185	91%	6623.65	580
3	187	92%	6551.65	580
4	189	93%	6513.8	580
5	191	94%	5716.15	540
6	193	95%	6248.5	570
7	195	96%	6370.45	580

Note: scenario 1 is the base scenario.

**Table 8:** Details of model I and model II.

Model	Objective function	Constraints	Features/differences
Model I	Formula (1)	Formulas (2)–(16)	Consider priority constraints
Model II	Formula (1)	Formulas (2) and (6)–(16)	Regardless of priority, parameter setting does not consider the nature of priority

**Table 9:** Parameters and results under three scenarios.

Scenarios	(*α*_*i*_, *β*_*i*_)			Revenue	Admission	Proportion
1	(0.9, 0.5)	(0.2, 0.1)	(0.1, 0)	7138.1	586	89.76%, 10.07%, 0.17%
2	(0.7, 0.5)	(0.3, 0.1)	(0.1, 0)	6815.55	583	69.64%, 29.33%, 1.03%
3	(0.7, 0.5)	(0.3, 0.1)	(0.1, 0.05)	6673.95	580	70.00%, 20.00%, 10.00%

## Data Availability

The data used to support the findings of this study are restricted by Admission Service Center of West China Hospital in order to protect patient privacy. Data are available from West China Hospital for researchers who meet the criteria for access to confidential data.
